The article "Comprehensive Bioinformatics Analysis of Gasdermin Family of Glioma" was retracted in 2023. Reasons: signs of a paper mill; compromised peer review; unreliable results or conclusions.

# Comprehensive Bioinformatics Analysis of Gasdermin Family of Glioma

**DOI:** 10.1155/2022/9046507

**Published:** 2022-04-15

**Authors:** Huaduan Zi, Zhan Tuo, Qianyuan He, Jingshu Meng, Yan Hu, Yan Li, Kunyu Yang

**Affiliations:** Cancer Center Union Hospital Tongji Medical College, Huazhong University of Science and Technology, Wuhan 430022, China

## Abstract

Pyroptosis is a programmed cell death mediated by gasdermins (GSDMs). The prognostic value of pyroptosis-related genes in different tumor types has been gradually demonstrated recently. However, the prognostic impact of GSDMs expression in glioma remains unclear. Here, we present a comprehensive bioinformatic analysis of gasdermin family member gene expression, producing a prognostic model for glioma and creating a competing endogenous RNA (ceRNA) network. The mRNA expression profiles and clinical information of glioma patients were downloaded from TCGA and CGGA. A risk score based on the gasdermin family was constructed in the TCGA cohort and validated in CGGA. The Jurkat cell was used to verify the relationship between pyroptosis and activation-induced cell death (AICD). We identify a significant association between the expression of GSDMD and GSDME and the glioma stage. The least absolute shrinkage and selection operator (LASSO) Cox regression analysis was used to construct a prognostic gene model based on the four prognostic gasdermin family genes (GSDMC, GSDMD, GSDME, and PJVK). This model was able to predict the overall survival of glioma patients with high accuracy. We show that gasdermin family genes are expressed primarily by immune cells, endothelial cells, and neuronal cells in the tumor microenvironment, rather than by malignant tumor cells. T cells were significantly activated in high-risk patients; however, the activation-induced cell death (AICD) pathway was also significantly activated, suggesting widespread expiration of cytotoxic T lymphocytes (CTLs), facilitating tumor progression. We also identify the lncRNA/miR-296-5p/GSDMD regulatory axis as an important player in glioma progression. We have conducted a comprehensive bioinformatic analysis identifying the importance of gasdermin family members in glioma; a prognostic algorithm containing four genes was constructed.

## 1. Introduction

Glioma is the most common and deadly tumor of the central nervous system in adults [1]. Molecular research in glioma has advanced substantially; modern molecular classification is now combined with traditional histological classification to optimize glioma diagnosis, patient prognostication, and prediction of treatment response [2–4]. However, these classification systems do not fully resolve individual patient variation and are therefore suboptimal in providing risk stratification for glioma patients. Integration of further data is therefore required, with gene expression profiling representing a leading candidate method for further improving glioma classification [5].

The article "Comprehensive Bioinformatics Analysis of Gasdermin Family of Glioma" was retracted in 2023. Reasons: signs of a paper mill; compromised peer review; unreliable results or conclusions.

In 2015, pyroptosis was defined as a gasdermin-mediated programmed death process [6, 7]. The gasdermin superfamily (GSDMs) consists of human gasdermin A/B/C/D (GSDMA/B/C/D), gasdermin E (GSDME, also known as DFNA5), and DFNB59 (Pejvakin, PJVK; in mice by Gsdma1-3, Gsdmc1-4, Gsdmd, Dfna5, and Dfnb59) [8]. Among these conserved proteins, GSDMD and GSDME are the most studied in pyroptosis. With the exception of PJVK, all of these proteins have two conserved domains: the N-terminal pore-forming domain (PFD) and the C-terminal repressor domain (RD) [7]. The PFD of most gasdermins can induce pyroptosis, which PJVK has not detected. In general, gasdermins maintain oligomerization through the interaction between PFD and RD, and RD can inhibit the cytotoxic effect of PFD. When the host is stimulated by a variety of exogenous or endogenous factors, GSDMs are cleaved by caspases or granzymes, the N-terminal PFD is dissociated from the C-terminal RD, and the N-terminal PFD is then oligomerized and deposited in the cell membrane. Pores are formed on the cell surface leading to the release of inflammatory molecules and cell pyroptosis. Early studies identified that pyroptosis mainly occurs in macrophages; in a study of mouse macrophage treatment with anthrax lethal toxin, Friedlander demonstrated rapid release of cell contents and cellular death [9]. Gasdermin proteins have been linked to human diseases in the scientific literature; however, the specific mechanisms by which gasdermin proteins play a role in disease processes are poorly understood.

As a new form of programmed cell death, pyroptosis has recently been identified to play a dual role in tumor development and therapeutic response. The relationship between pyroptosis and cancer is complex: though pyroptosis can inhibit tumor development and progression, it can also result in a protumorigenic microenvironment that provides nutrients for cancer growth [10]. Recent study identified novel pyroptosis-related gene signatures associated with prognosis in ovarian and lung cancer [11, 12]. However, these gene sets primarily comprise inflammasome-related genes. GSDMs are the effectors of cell pyroptosis. In vitro investigations have demonstrated that gasdermin activation induces cell death in glioma cells [13]. However, gliomas comprise both malignant cells and non-tumor cells, such as stromal and immune cells. These non-malignant populations dilute the purity of glioma cells and play an important role in tumor biology [14]. When studying the effects of gasdermin family members on glioma in tumor specimens, attention should be paid to its expression distribution among different cell types within the tumor microenvironment. At present, no research has systematically characterized the relationship between the gasdermin family on the prognosis and the clinical characteristics of glioma.

The article "Comprehensive Bioinformatics Analysis of Gasdermin Family of Glioma" was retracted in 2023. Reasons: signs of a paper mill; compromised peer review; unreliable results or conclusions.

In the present study, we perform bioinformatic analysis to characterize the expression of gasdermin family members in glioma patients. We utilize The Cancer Genome Atlas (TCGA) and the Chinese Glioma Genome Atlas (CGGA) RNA sequencing data sets to investigate the relationship between gasdermin gene expression profiles, comparing these to patient survival. We use the least absolute shrinkage and selection operator (LASSO) to develop four genetic risk characteristics. We character the relationship between this risk score and clinical characteristics of glioma patients. The single-cell RNA-seq (scRNA-seq) results demonstrate that the expression of gasdermins is mainly confined to monocytes/macrophages and CD8+ T cells. Gene set variation analysis (GSVA) showed that gasdermins are significantly related to the AICD pathway of T cells. Western blot results showed that antigen treatment could significantly activate the caspase-1/GSDMD pathway and induce T cells to pyroptosis. We also construct an mRNA-miRNA-lncRNA interaction network to clarify the potential molecular mechanism of GSDMD in glioma. This study is the first integrative study characterizing the role of GSDMs expression and its impact on clinical and molecular features of glioma.

## 2. Result

### 2.1. Relationships of GSDMs Expression with Clinical and Molecular Characteristics, Mutation Landscape, and Tissue Localization in Glioma

Six genes in the GSDM family were analyzed using the glioma transcriptome data from TCGA and CGGA. The results showed that GSDMD and GSDME were highly expressed in gliomas relative to GSDMA, GSDMB, GSDMC, and PJVK, and there was a significant correlation between them. For GSDMD, expression was significantly higher in WHO IV than in WHO II and III (Figure 1(a)). Protein-protein interaction (PPI) network demonstrated that genes related to pyroptosis interacted with one another, and the GSDMD is a hub gene with the local clustering coefficient was 0.625 (Figure 1(b)).  Figure 1(c) shows the position of CNV changes within these six genes on the respective chromosome. GSDM family genes were common targets of copy number amplification and deletion (Figure 1(c)). The frequency of mutation in GSDMA, GSDMB, GSDMC, GSDMD, GSDME, and PJVK were 0.4%, 0.1%, 3%, 3%, 0.6%, and 0.5%, respectively (Figure 1(d)), and the main genomic aberrations type is amplification. Both amplification and deep deletion events were observed in GSDMD, while both amplification and missense mutation events were identified in GSDMC (Figure 1(d)). In order to determine the source cell type of GSDM family gene expression within glioma tissue, we analyzed single-cell RNA-seq (scRNA-seq) data sets ((GSE89567, GSE102130, GSE103224, and GSE135437)). This identified monocytes/macrophages, T cells, and neurons as the major GSDM-expressing cell types, with low expression in malignant cells (Figure 1(e)).

The article "Comprehensive Bioinformatics Analysis of Gasdermin Family of Glioma" was retracted in 2023. Reasons: signs of a paper mill; compromised peer review; unreliable results or conclusions.

### 2.2. TMB, Drug Sensitivity Analysis, and Prognostic Impact of GSDMs

We first analyze the relationship between TMB and GSDMs (Figure 2(a)). Temozolomide (TMZ) is an oral alkylating agent that can cross the blood-brain barrier to reach the foci. It is one of the first-line, commonly used drugs in clinical chemotherapy for gliomas [15]. Next, we analyzed the relationship between gasdermin gene expression and the therapeutic sensitivity of temozolomide. There was a positive correlation between GSDMD and TMZ sensitivity (Figure 2(b)). The Pearson coefficient between GSDMD expression value and TMZ IC50 in different cell lines was −0.165 (*P* < 0.05). Then we analyzed the prognostic value of gasdermin family by univariate Cox regression analysis and analyzed prediction accuracy for one-, three-, and five-year survival by ROC analysis. The survival of glioma patients with high GSDMA expression was poor (Figure 2(c); *p* = 0.0042); similarly, survival time was low in patients with high expression of GSDMD (Figure 2(f); *p* < 0.0001) and GSDME (Figure 2(g); *p* = 0.00027). Conversely, low GSDMC expression was associated with poor survival (Figure 2(e); *p* = 0.00051). ROC curve analysis demonstrated our model had good predictive efficacy (GSDMA: AUC = 0.64 for one-year, 0.56 for two-year, and 0.52 for three-year survival; GSDMC: AUC = 0.63 for one-year, 0.61 for two-year, and 0.55 for three-year survival; GSDMD: AUC = 0.78 for one-year, 0.75 for two-year, and 0.68 for three-year survival; and GSDME: AUC = 0.61 for one-year, 0.61 for two-year, and 0.54 for three-year survival; Figure 2(c)–2(h)).

### 2.3. Construction of a Prognostic Model

The prognostic models by six genes in the GSDM family were constructed by LASSO Cox regression analysis.  Figure 3(a) shows the general situation of LASSO coefficients of six genes.  Figure 3(b) shows plots of the tenfold cross-validation error rates. Risk score = (0.2483) *∗* GSDMC + (0.7607) *∗* GSDM-D + (0.1264) *∗* GSDME + (−0.2989) *∗* PJVK. According to the risk score, glioma patients were divided into two groups. The risk score distribution, survival status, and the expression of four genes are shown in Figure 3(c). The increased risk score was associated with shorter survival time and increased risk of death (Figure 3(c)). Besides Kaplan–Meier analysis revealed poorer survival in patients with higher-risk scores compared to lower-risk scores (median time = 5.2 years vs. 10.3 years; *p* = 5.21e-07; Figure 3(d)), with AUCs of 0.819, 0.789, and 0.672 for the 1-, 3-, and 5-year ROC curves, respectively (Figure 1(d)).

The article "Comprehensive Bioinformatics Analysis of Gasdermin Family of Glioma" was retracted in 2023. Reasons: signs of a paper mill; compromised peer review; unreliable results or conclusions.

Finally, we harnessed two glioma patient data sets of CGGA to demonstrate the association between high-risk score and shorter survival. Then the CGGA data of 301 cases and 325 cases also revealed that glioma patients with high-risk scores had a worse overall survival probability than those with low-risk scores (Figures 3(e) and 3(f)). At the same time, we found that risk score can well predict the prognosis and recurrence of radiotherapy in patients with LGG (Figures S2 and S3). But in GBM, the prediction effect of the model was not satisfying (Figure S1).

### 2.4. Risk Score in relation to Clinical and Molecular Characteristics, Mutations, and Methylation in Glioma

Next, we explored differences in risk scores according to molecular and pathological characteristics of glioma. Higher-risk score was associated with higher histopathological glioma grade (Figures 4(a)–4(c)). The classical and mesenchymal subtypes of glioma demonstrated higher-risk scores (Figures 4(d) and 4(e)). ROC analysis was used to evaluate the ability of the risk score to distinguish the classical and mesenchymal cell subtypes in glioma. The ROC AUC was 86.6% and 89.2% in the TCGA and CGGA cohorts, respectively (Figures 4(d) and 4(e)). These data suggest a potentially important role for the calculated risk score in glioma progression. The risk score may also serve as a biomarker for the classical subtype. The risk score for WHO IV was higher than that of WHO II and III (Figure 4(f)). Moreover, the risk score of IDH wild-type cases was higher than those with IDH mutation (Figure 4(g)); cases with chromosome 1p/19q non-codeletion also demonstrated a higher-risk score. The unmethylated MGMT cases also demonstrated a higher-risk score (Figures 4(h) and 4(i)).

Together, these data show that glioma patients in the wild-type IDH, 1p/19q non-codeletion, unmethylated MGMT, and WHO IV groups have higher-risk scores. This is consistent with the poor prognosis reported in IDH wild-type cases and relatively favorable outcomes of patients with 1p/19q codeletion or MGMT methylation [16–18].

### 2.5. The Relationship between Risk Score and Immune Infiltration

We further explored the relationship between risk score and immune infiltration within the tumor. We first calculated the ssGSVA scores of all kinds of immune cells in glioma tissues. Patients were divided into high- and low-risk groups according to the risk score. The burden of the major immune cell types DCs, B cells, and T cells in the tumor microenvironment was associated with high-risk scores (Figure 5(a)). The stromal score, immune score, and ESTIMATE score were determined using on the TCGA cases. There were apparent correlations between the risk score and stromal, immune, and ESTIMATE scores (Figure 5(b)). Spearman's correlation analysis demonstrated significantly correlation between the risk score and immune contexture (*r* = 0.6; *p* < 2.2*e* − 16), stromal contexture (*r* = 0.59; *p* < 2.2*e* − 16), and ESTIMATE score (*r* = 0.62; *p* < 2.2*e* − 16; Figure 5(b)).

The article "Comprehensive Bioinformatics Analysis of Gasdermin Family of Glioma" was retracted in 2023. Reasons: signs of a paper mill; compromised peer review; unreliable results or conclusions.

Next, we analyzed the correlation between risk score and immune checkpoint molecules such as PD1, PD-L1, PD-L2, CTLA4, LAG3, and IDO1. We identified significant positive correlations between the risk score and immune checkpoint molecules (Figure 5(c)). We then confirmed the relationship between GSDMs and T cell immune response in gliomas using GSVA analysis. We identified a positive correlation with T cell activation via T cell receptor contact with antigen bound to MHC molecule on antigen-presenting cell. An important result that emerged from the data was that the GSDMs gene is involved in activation-induced cell death (AICD) of T cells (Figure 5(d)), which plays an important role in T-cell tolerance [19]. Flow cytometry showed that Jurkat treated with cell fragments could significantly induce the increase of Annexin-V-PI+ cells. This suggests that antigen stimulation may induce pyroptosis of Jurkat cells. Furthermore, using western blot detection, we found that antigen stimulation could significantly induce the activation of the caspase-1/GSDMD pathway in Jurkat cells (Figures 5(e) and 5(f)). Next, we will select the genes with risk score correlation coefficient *R* > 0.5 for gene enrichment analysis; 1,163 genes were identified in TCGA; and 755 genes were identified in the CGGA set for gene ontology analysis (Figure 5(g)). The results showed that high-risk score was significantly correlated with immune response, neutrophil activation, and T cell activation, alongside other pathways (Figure 5(h)).

### 2.6. Risk Score Is Associated with Different Patterns of Genomic Changes

The TCGA data set was investigated for patterns of genomic changes according to risk score: cases were divided into high- and low-risk scores. Mutation frequency comparison revealed higher numbers of somatic mutations in the high-risk score cases. Mutations in IDH1, CIC, FUBP1, and NOTCH1 were significantly enriched in the low-risk score cases. High-risk score cases demonstrated more frequent mutation of PTEN and NF1. Significant differences in TTN MUC16 FLG RYR2 LRP2 and SPTA1 mutations were also detected under various conditions with high-/low-risk scores (Figures 6(a) and 6(b)). Next, we studied the changes of somatic cell copy number between patients with low- and high-risk scores. As shown in Figure 6(c), gliomas with higher-risk score demonstrated frequent Chr7 amplification and Chr10 deletion (Figure 6(c)). However, the incidence of 1p/19q codeletion, as a genomic marker of oligodendroglioma, decreased with the increase of risk score expression in gliomas. We also examined the correlation between risk score and genome variation. As the results show, risk score is positively correlated with TMB, fraction genome altered, and aneuploidy score (Figure 6(d)).

The article "Comprehensive Bioinformatics Analysis of Gasdermin Family of Glioma" was retracted in 2023. Reasons: signs of a paper mill; compromised peer review; unreliable results or conclusions.

### 2.7. Building a Predictive Nomogram

We established a predictive nomogram (nomogram) to predict survival probability. Univariate and multivariate analysis showed that GSDMA and GSDMD expressions were independent factors affecting the prognosis of glioma patients (Figure 7(a)). Compared with the ideal model in the whole queue, the one-, three-, and five-year overall survival rate can be predicted with good efficacy compared using the prognostic nomogram (Figures 7(b) and 7(c)).

### 2.8. Construction of a Network of mRNA-miRNA-lncRNA

In order to clarify the potential molecular mechanism of GSDMD in glioma, we constructed an mRNA-miRNA-lncRNA interaction network. We identified four miRNAs as target mRNAs bound to GSDMD according to miRDB and starBase (Figure 8(a)). Among them, hsa-miR-296-5p demonstrated the highest target score; we therefore explored its upstream lncRNA target to construct the miRNA-lncRNA axis. Four lncRNAs (KCNQ1OT1, LINC01278, MIRLET7BHG, and NEAT1) were identified as target lncRNAs (Figures 8(b) and 8(e)). A ceRNA network was visualized; KCNQ1OT1 and LINC01278 were positively correlated with glioma staging, while MIRLET7BHG and NEAT1 were negatively correlated with staging (Figure 8(c)). Survival analysis demonstrated that high LINC01278 and MIRLET7BHG were associated with better prognosis, while NEAT1 was associated with poorer survival (Figure 8(d)). There was no significant association between KCNQ1OT1 and survival.

## 3. Conclusion

In the present study, we perform bioinformatic analysis to characterize the expression of gasdermin family members in glioma patients. We utilize The Cancer Genome Atlas (TCGA) and the Chinese Glioma Genome Atlas (CGGA) RNA sequencing data sets to investigate the relationship between gasdermin gene expression profiles, comparing these to patient survival. We use the least absolute shrinkage and selection operator (LASSO) to develop four genetic risk characteristics. We character the relationship between this risk score and the clinical characteristics of glioma patients. The single-cell RNA-seq (scRNA-seq) results demonstrate that the expression of gasdermins is mainly confined to monocytes/macrophages and CD8+ T cells. Gene set variation analysis (GSVA) showed that gasdermins are significantly related to the AICD pathway of T cells. Western blot results showed that antigen treatment could significantly activate the caspase-1/GSDMD pathway and induce T cells to pyroptosis. We also construct an mRNA-miRNA-lncRNA interaction network to clarify the potential molecular mechanism of GSDMD in glioma. This study is the first integrative study characterizing the role of GSDMs expression and its impact on clinical and molecular features of glioma.

The article "Comprehensive Bioinformatics Analysis of Gasdermin Family of Glioma" was retracted in 2023. Reasons: signs of a paper mill; compromised peer review; unreliable results or conclusions.

## 4. Discussion

Pyroptosis can release inflammatory factors and stimulate normal cells to induce malignant transformation [20]. Conversely, pyroptosis can promote the immunogenic death of tumor cells and activate anti-tumor immunity, making it a potential prognostic and therapeutic target for cancer [20]. In ovarian cancer and lung cancer, a new PRG signature has been identified to predict prognosis [11, 12]. However, the role of PRG in glioma is not yet clear; we aim to dissect the role of PRG in this disease context.

Glioma is composed of both immune cells and stromal cells, alongside malignant tumor cells. Microglia are non-malignant myeloid-derived cells found in the brain parenchyma; these cells can produce macrophage-like reactions under pathological conditions [21]. Large numbers of microglia have been found within glioma masses, and the degree of microglial infiltration has been positively associated with the degree of glioma malignancy [22, 23]. Previous studies have focused on the pyroptosis of malignant cells themselves without considering the impact of pyroptosis in non-malignant cells in the tumor microenvironment. GSDME has been shown to play an important role in the toxic and side effects of chemotherapy drugs on normal tissues [24]. It has been suggested that GSDME-mediated pyroptosis of macrophages is the key pathological mechanism of cholestatic liver injury [25].

Immune cell pyroptosis was first discovered in monocytes/macrophages and is an important form of immune cell death. Therefore, when exploring the impact of PRG in glioma, its “tissue specificity” must be considered. We demonstrate that gasdermin family genes are mainly expressed in immune cells rather than tumor cells. We also identify a large number of aggregates in endothelial and neuronal cells. We show that GSDME expression is low in most tumor cell lines due to GSDME gene promoter methylation, while GSDME is widely expressed in cell lines representing normal tissues [24]. In Gsdme-/- mice, intraperitoneal injection of cisplatin or 5-FU leads to immune cell infiltration and severe intestinal damage [26]. In addition, flagellin AN/C inhibits radiation-induced ROS production in intestinal epithelial cells reduces NLRP3 activity and ultimately inhibits caspase-1-dependent pyroptosis, which may be an important factor in protecting intestinal epithelial cells from radiation damage [27]. Of course, many studies have revealed that GSDMs promotes the occurrence of anti-tumor immunity and has a beneficial effect [28, 29].

The article "Comprehensive Bioinformatics Analysis of Gasdermin Family of Glioma" was retracted in 2023. Reasons: signs of a paper mill; compromised peer review; unreliable results or conclusions.

In this study, we first explored the expression and prognostic value of gasdermin family genes in glioma. We identified a positive correlation between GSDMD and GSDME expression and glioma staging. Prognostic analysis suggested a poor survival rate in glioma patients with low expression of GSDMC and high GSDMD or GSDME expression. LASSO Cox regression analysis was used to construct a prognostic gene model based on four prognostic gasdermin family member genes (GSDMC, GSDMD, GSDME, and PJVK); the model was able to predict the overall survival of patients with glioma with medium to high accuracy. The forecast nomogram shows that the three- and five-year overall survival rates can be predicted relatively well compared to the ideal model in the entire cohort. However, this model is not suitable for glioblastoma multiforme (GBM). Previous studies have identified that autophagy and ferroptosis-related prognostic signatures perform well in predicting the prognosis of GBM patients [30, 31]. In our research, we first determined the prognostic gene characteristics of the gasdermin family of glioma, which provides more options for the prognosis prediction of LGG.

We further explored the relationship between this model and the clinical features of glioma. A high-risk score is related to the degree of malignancy, such as a high WHO level. In addition, the risk score was higher in the mesenchymal glioma subtype. This subtype is characterized by mesenchymal differentiation and NF1 mutation and demonstrates poor immune engagement and aggressive clinical behavior. This is the first study to present the expression pattern of gasdermin family members in gliomas according to the WHO classification system, TCGA subtype, or 2016 WHO molecular classification [32]. In this study, we investigated different genomic changes according to the risk score. We identified somatic mutations and CNA events correlated with a differential risk score. In cases with high-risk scores, oncogenic drivers such as mutations in EGFR, PDGFRA, PIK3C2B, and CDK4 were detected at different frequencies.

The article "Comprehensive Bioinformatics Analysis of Gasdermin Family of Glioma" was retracted in 2023. Reasons: signs of a paper mill; compromised peer review; unreliable results or conclusions.

In the gene ontology analysis of biological functions, we found that risk score is significantly correlated with the infiltration of various immune cell types. Moreover, numerous immune checkpoint molecules were highly expressed with increasing risk scores. We also calculated the GSVA score of T cell-related pathways to explore the relationship between risk and T cell function. This analysis identified that while T cells are significantly activated in the high-risk group, the AICD pathway was also activated. This may represent one mechanism by which CTLs are inactivated within this patient group in order to facilitate tumor progression. We found for the first time that antigen stimulation can significantly induce the activation of the caspase-1/GSDMD pathway in tumor cells. This provides a new idea for the mechanism of AICD.

Cancer immunotherapy has demonstrated marked efficacy in some clinical contexts. Clinical trials of immune checkpoint blocking for gliomas are ongoing [33]. Many investigators have posited that TMB-based detection methods can help identify patient groups that respond to immunotherapy [34–36]. However, this detection method has not achieved optimal predictive power in glioma [37]. Our findings suggest that this may be due to immune cells with gliomas of the high TMB group, which is rich in GSDMs member expression, which are prone to AICD, which in turn modules sensitivity to immunotherapy.

We also constructed an mRNA-miRNA-lncRNA network. We found that KCNQ1OT1/LINC01278/MIRLET7BHG/NEAT1 can be used as the upstream target of miR-296-5p to regulate the progression of glioma. Studies have found that silencing KCNQ1OT1 reduces pyroptosis by targeting miR-214-3p and caspase-1 [38]. Neat1 is associated with NLRP3, NLRC4, and AIM2 inflammasomes in mouse macrophages to enhance their assembly and subsequent pro-caspase-1 processing [39, 40]. Our research suggests for the first time that NEAT1 may directly regulate the expression of GSDMD through has-miRNA-296-5p and thus affect cell pyroptosis. Further research is required to independently confirm these findings.

In summary, our study investigated the biological significance of gasdermin family genes using large cohorts of glioma cases. Our findings indicate that gasdermin family members may serve as important biomarkers within glioma, and their expression is associated with differences in tumor mutation spectrum, copy number events, histology, and clinical features.

The article "Comprehensive Bioinformatics Analysis of Gasdermin Family of Glioma" was retracted in 2023. Reasons: signs of a paper mill; compromised peer review; unreliable results or conclusions.

## 5. Method

### 5.1. Data Collection

The 698 glioma samples within the TCGA RNA-seq database were accessed (https://portal.gdc.cancer.gov/) and used as a training cohort. The CGGA RNA sequencing (RNA-seq) data set (mRNAmicroarray_301 and mRNAseq_325) and corresponding clinical and molecular information were retrieved for use as a validation set. We used TCGA and CGGA original data, wherein 60,483 genes were detected in TCGA database and 19,416 genes were detected in CGGA database. Cases with mismatching identifiers between the transcriptome data and clinical annotation were removed prior to analysis. The RNA-seq data of specific tumor anatomy in GBM identified by H&E staining were retrieved from the Ivy Glioblastoma Atlas Project (https://glioblastoma.alleninstitute.org/). Drug-sensitivity-related data were obtained from the Cancer Cell Line Encyclopedia (https://sites.broadinstitute.org/ccle).

### 5.2. Mutation Analysis of Gasdermin Family Gene

Corresponding somatic mutation and copy number alteration (CNA) data for samples were accessed through the TCGA database. The mutation frequencies of gasdermin family genes and corresponding oncoplot/waterfall plots in LGG patients were generated using the “maftools” package. CNA positions on chromosome 23 were mapped using the “RCircos” package.

### 5.3. Development of the Prognostic Model

Raw RNA-sequence data (level 3) and corresponding clinical annotation for the CC tumors were obtained from The Cancer Genome Atlas (TCGA) database (https://portal.gdc.com). Survival differences were analyzed using the log-rank test. Time ROC analysis was used to compare the prediction accuracy and risk score of the XX gene. The least absolute shrinkage and selection operator (LASSO) regression algorithm was used for feature selection. Tenfold cross-validation was implemented to assess the model. The above analysis was implanted using the glmnet package in *R*.

For Kaplan–Meier survival curves, the hazard ratio (HR) and 95% confidence interval (CI) were obtained by univariate Cox proportional hazard regression models. All of the above analysis methods and *R* software packages are implemented using v4.0.3 *R* software (R Foundation for Statistical Computing, 2020). A threshold of *p* < 0.05 was considered statistically significant.

### 5.4. Competing Endogenous RNA Network Construction

To clarify the potential function of GSDMD in LGG, we constructed a competitive endogenous RNA (ceRNA) network. StarBase (https://starbase.sysu.edu.cn/) and MiRDB (https://mirdb.org/) were used to predict miRNA targets. Based on the identified miRNA, StarBase (https://starbase.sysu.edu.cn/) and LncBase Predicted v2 (https://carolina.imis.athena-innovation.gr/diana_tools/web/index.php?r=lncbasev2/index-predicted) were used to predict the lncRNA target that interacts with miRNA. We also used the TCGA data set to explore the expression and prognostic value of these miRNA and lncRNA targets. All analyses were considered statistically significant when *p* < 0.05.

The article "Comprehensive Bioinformatics Analysis of Gasdermin Family of Glioma" was retracted in 2023. Reasons: signs of a paper mill; compromised peer review; unreliable results or conclusions.

### 5.5. Cell Lines and Antibodies

The Jurkat and U251 glioma tumor cell line were obtained from the American Type Culture Collection and were cultured with RPMI-1640 with 10% fetal bovine serum (Gibco). The following primary antibodies were used: anti-caspase-1 (abclonal), anti-GSDMD (Sigma), and anti-GAPDH (abclonal).

### 5.6. Western Blot Analyses

Cultured cells were washed twice with ice-cold PBS, and total protein extraction was performed using RIPA lysis buffer containing 1 mmol/L phenylmethanesulfonyl fluoride (PMSF) together with protease and phosphatase inhibitors. Cytosolic protein, nuclear protein, and membrane protein extraction were performed according to the manufacturer's protocol. The protein concentration was then determined by the Bradford method using bovine serum albumin (BSA, 0.1 mg/mL) as the standard. Equal concentrations (30 mg) of total protein were subjected to 10% polyacrylamide SDS gel electrophoresis and transferred to PVDF membranes. The membranes were blocked with 5% skim milk in Tris-buffered saline containing Tween (TBST) buffer (10 mmol/L Tris-HCl (pH 7.4), 150 mmol/L NaCl, and 0.1% Tween-20) for 2 h. Protein expression was detected using primary antibodies incubated overnight at 4°C, followed by incubation with secondary antibodies for 1 h at RT. After the membranes were washed with TBST buffer 3 times, the proteins were visualized with enhanced chemiluminescence reagent.

### 5.7. Statistical Analysis

R language (v3.6.3), SPSS software (v22.0), and GraphPad Prism (v8.0) for Windows were used for statistical analyses and generating figures. All error bars in graphical data represent the mean ± SE. Spearman's rank correlation was used to analyze the association. The Student's two-tailed *t*-test and the Wilcoxon test were used to determine the statistical relevance between groups, and *p* < 0.05 was considered significant.

## Figures and Tables

**Figure 1:** Expression profile and mutation landscape of GSDMs in glioma: (a) expression of gasdermins in different WHO grades through different databases, (b) PPI network showing the interactions of the GSDMs, (c) the location of CNV alterations of GSDMs on chromosomes, (d) the mutation frequency and classification of GSDMs in glioma, and (e) single-cell RNA-seq were enrolled to determine the location of GSDMs in different cell types.

The article "Comprehensive Bioinformatics Analysis of Gasdermin Family of Glioma" was retracted in 2023. Reasons: signs of a paper mill; compromised peer review; unreliable results or conclusions.

**Figure 2:** TMB, drug sensitivity analysis, and prognosis of GSDMs: (a) the correlation between GSDMs and TMB, (b) the correlation between GSDMs and chemotherapeutic drug sensitivity, and (c)–(h) relationship between the six genes and prognosis in gliomas.

**Figure 3:** Construction of a prognostic model: (a) LASSO regression analysis chart; (b) LASSO regression cvfit chart; (c) distribution of risk score, survival status, and the expression of GSDMs; and (d)–(f) overall survival curves for glioma patients in the high-/low-risk group and the ROC curve of measuring the predictive value in different data sets.

**Figure 4:** The outlook of clinical and molecular features in associations with risk score: (a)–(c) the risk score in different histopathologic classification by different data sets (A: strocytoma, O: oligodendroglioma, AO: Anaplastic oligodendro, AA: anaplastic astrocy-toma, pGBM: primary glioblastoma, sGBM: secondary glioblastoma, and rGBM: recurrence of pGBM). (d) and (e) the risk score in molecular subtype. ROC curves predicted GSDMs as a biomarker of classical subtype glioma. (f) The risk score increases by the WHO grade. (g) Risk score was upregulated in the IDH wild-type gliomas compared with the IDH mutant gliomas. (h) The 1p/19q non-codeletion of GSDMs has a higher risk score than the codeletion. (i) The risk score of unmethylated group was higher than that of methylated group.

**Figure 5:** Risk score is related to tumor immune infiltration: (a) risk score varies among many immune cells, (b) tumor microenvironment score was significantly correlated with risk score, (c) relationship between risk score and immune checkpoint, (d) high-risk score indicates the enrichment of AICD pathway, (e) Jurkat treated with cell fragments could significantly induce the increase of Annexin-V-PI+ cells, (f) antigen stimulation significantly induces the activation of caspase-1/GSDMD pathway, and (g) relationship between risk score and gene enrichment analysis.

**Figure 6:** Distinct genomic profiles associated with the risk score: (a) and (b) differential somatic mutations were detected in gliomas with low- and high-risk score, (c) the overall CNAs profile in order of upregulation of risk score, and (d) correlation between risk score and TMB, fraction genome altered, aneuploidy score, and MSI mantis score.

**Figure 7:** Construction of a predictive nomogram: (a) hazard ratio and *p*-value of the constituents involved in univariate and multivariate Cox regression and (b) and (c) nomogram to predict the one-, three-, and five-year overall survival rate of glioma patients. Calibration curve for the overall survival nomogram model in the discovery group. A dashed diagonal line represents the ideal nomogram.

The article "Comprehensive Bioinformatics Analysis of Gasdermin Family of Glioma" was retracted in 2023. Reasons: signs of a paper mill; compromised peer review; unreliable results or conclusions.

**Figure 8:** Construction of ceRNA network: (a) results of miRNA target predicted by mirTarBase and TarBase V8, (b) results of lncRNA targets predicted by lncBase predicted V2 and StarBase V2.0, (c) the expression of four LncRNA in glioma, (d) the prognostic value of miR-335-5p in glioma, and (e) the network of lncRNA-miRNA-mRNA.

## Data Availability

The data could be download at https://portal.gdc.cancer.gov/, https://xenabrowser.net/, and https://www.cgga.org.cn/, and the codes used during the current study are available from the corresponding author on reasonable request.

## Abbreviations

ceRNA: Competing endogenous RNA
LASSO: Least absolute shrinkage and selection operator
AICD: Activation-induced cell death AICD
CTLs: Cytotoxic T lymphocytes CTLs
PFD: Pore-forming domain
RD: Repressor domain
TCGA: The Cancer Genome Atlas
CGGA: Chinese Glioma Genome Atlas
GSVA: Gene set variation analysis
scRNA-seq: Single-cell RNA-seq
DAC: Dexitabine
TMZ: Temozolomide
TMB: Tumor mutation burden
GBM: Glioblastoma multiforme
LGG: Lower-grade glioma.

## Supplementary Materials

Supplementary Materials Figure S1: evaluate the prognostic roles of risk score: (A) forest plot of the prognostic ability of the GSDMs in GBM and (B) and (C) Kaplan–Meier curves showing that the survival of the high score group is poor. Figure S2: risk score predicts a patient's prognosis after radiotherapy: (A) and (B) Kaplan–Meier curves showing that risk score was a good predictor of outcome in patients who received radiation therapy. Figure S3: risk score predicts the outcome of a patient's treatment: (A) and (B) high-risk score can predict new lesions after initial treatment and poor treatment outcomes in low grade glioma.
